The article "Deformation Analysis and Research of Building Envelope by Deep Learning Technology under the Reinforcement of the Diaphragm Wall" was retracted in 2023. Reasons: unreliable results or conclusions; concerns about the data; concerns about the results or conclusions; concerns about the peer review.

# Deformation Analysis and Research of Building Envelope by Deep Learning Technology under the Reinforcement of the Diaphragm Wall

**DOI:** 10.1155/2022/9489445

**Published:** 2022-09-14

**Authors:** Lijuan Wang, Qihua Zhao

**Affiliations:** State Key Laboratory of GeoHazard Prevention and GeoEnvironment Protection, Chengdu University of Technology, Chengdu 610059, China

## Abstract

The safety analysis of underground buildings is the most crucial problem in the construction industry. This work aims to optimize the safety analysis results of the underground building envelope and comprehensively improve the safety of the underground building. Long short-term memory (LSTM) can make long-term and short-term predictions, thus reducing the model's prediction error. Applying it to the deformation analysis, data prediction of the underground building envelope can improve the accuracy of the deformation prediction of the envelope. This work deeply discusses deep learning technology and the principle of the LSTM model. Based on the safety analysis concept of the underground building envelope, LSTM underground building envelope deformation's prediction model is established and comprehensively evaluated. The results show that in the prediction of horizontal displacement of foundation pit pile of diaphragm wall, the mean relative error (MRE) of the prediction results of the designed model range in 10%–18%, and the calculation time ranges 15–36 s. In the settlement displacement prediction, the model's MRE is within the range of 5%–7%, and the calculation time is within the range of 17–40 s. With the increase of training times, the prediction accuracy of the model increases, and the calculation time becomes relatively stable. Compared with other models, the relative error of prediction results is about 5.4% at the highest and 1.8% at the lowest. This work provides technical support for improving the safety prediction accuracy of the underground building envelope and provides some reference value for the comprehensive development of the underground building industry.

## 1. Introduction

With the change of society, the construction industry has become the basic force supporting social development. To continue healthy survival, human beings must protect the natural environment, reduce the amount of land occupied, and develop underground space, to effectively solve the problem of urban land shortage and maintain the sustainable development of the city [1]. In recent years, with the strong support of national policies, the domestic underground construction industry has developed steadily, but the underground construction industry also faces various problems along with opportunities [2]. Among them, the safety analysis of underground buildings is the most vital problem, and the construction of safety analysis models of underground buildings with excellent performance has become the main driving force for its progress. Deep learning (DL) technology, as a relatively mature artificial intelligence (AI) technology at present, has a good development prospect to build a safety analysis model of the underground building [3]. Although the current application of this technology is not perfect, many studies have provided technical support for it.

The long short-term memory (LSTM) network is a DL model based on the recurrent neural network (RNN). It inherits the recursive cycle and time sequence characteristics of RNN, effectively overcomes the gradient disappearance problem, and can realize information's long-term and short-term memory. In order to optimize the working mode of the pump station and reduce energy consumption, Lee and Lee established a neural network model based on LSTM to predict the energy consumption of the pump station. The results showed that the prediction had high accuracy and generalization ability [4]. Luo and Oyedele proposed a hybrid prediction model combining radial basis function neural network and LSTM neural network optimized by the tree-seed algorithm to improve the accuracy, robustness, and generalization of building energy consumption prediction [5]. Based on this, the envelope structure of underground buildings is first discussed, and the diaphragm wall's main structure is discussed. Then, the basic concepts of DL technology and its branch technologies are introduced. Finally, based on the deformation analysis of the underground building envelope, the long short-term memory (LSTM) underground building deformation prediction model is constructed. LSTM envelope prediction model mainly calculates the condition of the envelope structure through the LSTM algorithm and then predicts the envelope structure's deformation result. The research innovation is to apply the LSTM model to the deformation analysis of underground building envelope structures from the perspective of diaphragm wall reinforcement and further explore the comprehensive performance of the model under different training times. This exploration provides technical support for deformation analysis of underground building envelope and provides a reference for safety analysis and optimization of underground buildings. It provides a new method for improving the deformation prediction of the underground building envelope. It provides a reference for the optimization of underground buildings and promotes the comprehensive development of the underground construction industry.

### 1.1. Literature Review

Li et al. described and analyzed in detail the potential safety problems brought by underground buildings to fire safety work [6]. Zhi et al. made a detailed analysis of the factors affecting the comfort of the internal environment after the completion of urban underground buildings and analyzed the impact of urbanization on people's living environment. The relationship between the energy consumption of underground buildings and indoor temperature and humidity was further analyzed [7]. Wang et al. used the finite element numerical simulation method to study the instability of the subway foundation pit under the influence of heavy rainfall. According to the hydraulic coupling conditions caused by rainfall, a fluid-solid coupling numerical model of a large-scale deep foundation pit in Earth rock composite stratum was established [8]. Li et al. studied the theoretical relationship between DL and building detection and discussed the research on the detection and segmentation of changes in buildings, such as color and reflectivity of remote sensing images [9]. Based on the small strain hardening model of soil and the corresponding model parameters, Gao et al. conducted a three-dimensional finite element numerical simulation of the excavation process of the foundation pit and compared the lateral displacement of the foundation pit envelope structure and the surface settlement outside the pit with the field monitoring data [10]. According to life cycle cost analysis, Himmetoglu et al. used the EnergyPlus building performance simulation program, artificial neural network, and genetic algorithm to determine the most suitable green envelope design for buildings in earthquake areas with different climates [11]. Chen et al. used the optical fiber temperature measurement system to detect the position of the seepage point during the open-pit excavation of a station of Qingdao Metro. Through numerical calculation and field measurement, the abnormal change of the seepage field caused by the seepage point was obtained [12]. Wang et al. studied the influence of deep foundation pit excavation on foundation pit deformation in saturated soft loess areas through a field test on deformation characteristics of deep foundation pit in saturated soft loess areas with a high water level and clarified the deformation laws of foundation settlement, envelope structure, and supporting axial force [13]. DL adopts an unsupervised layer-by-layer training algorithm to realize the effective expression of data feature information and has strong nonlinear data fitting ability. DL realizes feature extraction from low-level to high-level for external input data by establishing a hierarchical structure simulating the human brain [14].

The research literature suggests that there are few studies on the deformation analysis of the envelope structure using the algorithm technology under the reinforcement of the diaphragm wall. LSTM is a network algorithm in the DL model. Its advantages are that it has the ability of self-learning, self-adaptation, and efficient memory. Besides, it has a strong fitting ability to highly nonlinear time-series data and can make long-term and short-term prediction, thus reducing the model's prediction error. The innovative application of the LSTM model to the deformation analysis data prediction of the underground building envelope can improve the prediction accuracy of envelope deformation [15].

## 2. Research Theory and Method

### 2.1. Underground Building Envelope

With the development of society, urban construction is also accelerating, but in the process, it is also necessary to protect the red line of arable land and the environment. Therefore, in the current urban construction, the construction of underground space is becoming more and more important. At present, the underground shopping malls, subway platforms, and underground parking lots in major cities are increasing day by day, and the construction of these underground projects must inevitably involve a large number of technical problems of foundation pit engineering. As the requirements of the city continue to change, foundation pit projects now have deeper, larger requirements, and more severe challenges such as poorer soil conditions and more complex surrounding built environments [16]. Therefore, more engineering problems arise to be solved and studied. At the same time, to solve the problem of urban traffic congestion, major cities have begun to vigorously develop subway light rail and other rail transportation. For the subway foundation pit, due to the construction in the city, the requirements for the displacement of the foundation pit and the settlement of the surrounding buildings are stricter, so the support scheme of it also puts forward higher requirements and restrictions [17]. The current underground building envelope is generally a combination of a diaphragm wall and steel plate, and this maintenance structure plays a momentous role in the development of underground buildings.  Figure 1 shows the basic principle of the composite envelope of the diaphragm wall and multiple rows of steel plates.

In Figure 1, the composite envelope of diaphragm wall and multiple rows of steel plates consists of three parts, namely diaphragm wall, multiple rows of steel sheet piles, and a top connecting plate. Among them, the diaphragm wall has the function of high rigidity, mainly acts as soil and water-retaining, and bears the horizontal load generated after the excavation of the foundation pit and the vertical load transmitted by part of the top. It is the main load-bearing member of the composite envelope and controls the horizontal deformation [18]. The function of the multirow steel sheet piles is that they are located behind the diaphragm wall and can share part of the horizontal load to play the role of assisting in resisting lateral movement, and at the same time, it can also assist in controlling the vertical deformation around the foundation pit. The function of the top connecting plate is to mainly coordinate the front and rear force and deformation and distribute the top load evenly to multiple rows of steel sheet piles and diaphragm wall. Simultaneously, a certain construction platform is formed, which can withstand a certain vertical load of the heavy-duty access road. It increases the external construction space of the foundation pit [19]. Preliminary analysis from the perspective of force and deformation shows that composite envelope has certain scientific and rationality. However, how to design the structure, its working properties, use effect, economic benefits, and application prospects in actual work still need to be deeply studied [20].

### 2.2. Reinforcement of Ground Walls

As the main part of the current composite envelope of the diaphragm wall and multiple rows of steel plates, the diaphragm wall is a kind of grooving machine used on the ground for the foundation project, along the peripheral axis of the deep excavation project, under the condition of mud wall protection, to excavate a long and narrow deep groove. After cleaning the groove, the steel cage is hung in the groove, and then the underwater concrete is poured into a unit groove section by the conduit method. In this way, a continuous reinforced concrete wall is built underground as a water interception, antiseepage, load bearing, and water-retaining structure [21]. According to the way of forming the wall, the diaphragm wall can be divided into pile row type, slot plate type, and combined type. According to the purpose of the wall, it can be split into an antiseepage wall, temporary retaining wall, and permanent retaining (load bearing). By the material of the wall, it can be divided into the reinforced concrete wall, plastic concrete wall, solidified mortar wall, self-hardening mud wall, prefabricated wall, mud groove wall, post-tensioned prestressed wall, and steel wall. From the excavation situation, it can be segmented into the underground retaining wall (excavation) and underground seepage prevention wall (without excavation) [22].

Due to the limitation of construction machinery, the thickness of the diaphragm wall has a fixed modulus and cannot be flexibly adjusted according to the diameter and stiffness of the pile like the cast-in-place pile. Hence, it can only show economical and unique advantages under a certain depth of foundation pit engineering or other special conditions. It is generally applicable to the following conditions: deep foundation pit projects with a depth of more than 10 meters; the envelope is also a part of the main structure and has strict requirements on waterproofing and impermeability; the reverse method is used for construction; and the ground and underground are synchronized. During construction, a diaphragm wall is generally used as the envelope wall; the space in the foundation pit is limited, the distance between the basement exterior wall and the red line is very close; and other enclosure forms cannot meet the operation requirements of the construction; in the ultradeep foundation pit, for example, 30 m–50 m deep foundation pit project, when other enclosures cannot satisfy the requirements, the diaphragm wall is often used as the envelope [23].

Since the diaphragm wall plays a critical supporting role in the underground building, it is a very reasonable and feasible strategy to reinforce the composite envelope through the diaphragm wall [24]. The principle of reinforcement of the composite envelope by the diaphragm wall is exhibited in Figure 2.

Figure 2 suggests that four kinds of reinforcement methods of diaphragm walls are currently widely used.

1. The first is the reinforcement method of advance precipitation in the pit. At first, this method was used to reduce the soil moisture content at the bottom of the foundation pit to provide conditions for excavation. At present, this method is mainly adopted to improve the poor foundation. The main principle is to reduce groundwater's height and improve the soil's strength through the dewatering well. After the strength of the soil is strengthened, the plasticity of the soft underlying soil layer is weakened, so that the overall strength is increased, and the deformation value of the soft muddy soil can be significantly reduced [25].
2. The second method is high-pressure jet grouting reinforcement, which is realized by combining the grouting pipe with the drill. First, the drill is adopted to drill to the ideal depth, that is, to drill to the formation position where shotcreting is required. Then, grouting is conducted to strengthen the diaphragm wall. The main principle of this method is to use the strong impact force of the fluid to recombine the cement slurry and the soft muddy soil, to improve the soil's strength, and then realize the reinforcement of the diaphragm wall. According to the different grouting processes, that is, according to the number of grouting pipes used in the grouting process, the grouting methods are divided into the single pipe, double pipe, and triple pipe methods [26].
3. The third method is cement-soil mixing reinforcement. Curing agents commonly used in cement-soil mixing and reinforcement include lime, cement, and other materials. The main method is to use the ultradeep mixer at the position of the weak stratum to directly mix the soil and several chemical curing agents at this position through strong mixing. When the chemical curing agent is mixed with the soil, it will react and make the soft soil become a whole with great strength. This method can improve the strength of the soft soil and the deformation stiffness of the soft soil layer. When the cement-soil mixing pile is adopted to improve the base soil mass, the entire diaphragm wall or other envelope structure will have a certain distance from the reinforcement body formed by cement soil. Hence, it cannot be closely connected and can only be supplemented by grouting or high-pressure jet grouting [27].
4. The fourth method is grouting reinforcement. The main process is to use the grouting pipe to uniformly distribute the slurry in the foundation of the muddy soft soil layer through high air pressure, liquid pressure, or electrochemical mechanism conditions to strengthen the foundation. The principle of this method is to fill, compact, and infiltrate the slurry into the soft soil particle structure to improve the foundation's strength and reinforce the diaphragm wall [28].

The above four methods are the most advanced methods to realize the reinforcement of the diaphragm wall through foundation reinforcement. The disadvantage of the third method is that it cannot be seamlessly connected with the support system, and general machinery has certain limitations in the reinforcement process. The second method usually has the problems of not being environmentally friendly and not economical. The last method is usually an uneven distribution of foundation strength after reinforcement is completed. Therefore, the method to use to reinforce the diaphragm wall also depends on the specific environment. This also exposes some obvious problems, the most serious of which is the deformation of the maintenance structure. It has an important impact on the safety of the underground building. So, it is the most reasonable decision to conduct research and analysis on it through technical means and solve the problem in time. From this, DL technology is used to focus on the problem of maintenance structure deformation under the reinforcement condition of the diaphragm wall, which provides a reference for the development of underground buildings.

### 2.3. DL Technology Model

DL technology is to learn the sample data's internal law and representation level. Its ultimate goal is to enable machines to have the same analysis and learning ability as people and to recognize data such as characters, images, and sounds. DL is a complex machine learning algorithm, and its effect in speech and image recognition is far more than the previous related technology [29]. The recurrent neural network (RNN) is one of the DL technologies. It is designed to use one of the RNN technologies to realize the research on the deformation analysis of the envelope structure under the condition of the diaphragm wall reinforcement [30].

LSTM is a special DL RNN technology, which is mainly adopted to solve the problems of gradient disappearance and gradient explosion in the process of long sequence training. Compared with ordinary RNN technology, LSTM can process longer sequences and performs better in long sequence task processing [31].  Figure 3 refers to the comparison effect of LSTM and common RNN techniques and the working principle of LSTM.

Figure 3 displays that LSTM is a DL model based on RNN technology, which fully possesses the characteristics of RNN technology and is also an optimization model of RNN technology. Its advantage lies in that, based on RNN technology, it can effectively overcome the problem of gradient disappearance and realize the long-term and short-term memory of information [32]. Each LSTM memory module contains one or more self-connected memory cells and three multiplication gates, which are input gate, forget gate, and output gate. The main role of the multiplication gate is to read, write, and reset the cell [33]. The three gate structures of the LSTM network can selectively memorize the input timing information and the correction parameters of the weights of each neuron in the backpropagation process and do not send their own behaviors as input or output values to other neurons. And only when the connection weight of the multiplication gate is 1, the corresponding data storage, reading, memory, and transmission operations can be performed. When the connection weight is 0, it does nothing. The calculation of the LSTM memory unit is as follows:

(1) $$\begin{array}{c} z^{f}=\sigma \left(w^{f}\cdot \left(\left[h^{t-1},x^{t}\right]\right)+b^{f}\right)\text{,}\\ z^{i}=\sigma \left(w^{i}\cdot \left(\left[h^{t-1},x^{t}\right]\right)+b^{i}\right)\text{,}\\ z^{o}=\sigma \left(w^{o}\cdot \left(\left[h^{t-1},x^{t}\right]\right)+b^{o}\right)\text{,} \end{array}$$

*z*^*f*^ represents the forget gate, *z*^*i*^ means the input gate, *z*^*o*^ expresses the output gate, *σ* refers to the activation function, generally tanh or “sigmoid”, *w* stands for the weight, and *b* denotes the paranoid term. There are also hidden neurons, which are calculated as

(2) $$\begin{array}{c} z=\sigma \left(w\cdot \left(\left[h^{t-1},x^{t}\right]\right)+b\right)\text{.} \end{array}$$

According to the above equation, the output result can be expressed as

(3) $$\begin{array}{c} c^{t}=z^{f}⊙c^{t-1}+z^{i}⊙z\text{,}\\ h^{t}=z^{o}⊙\tanh\;\left(c^{t}\right)\text{,}\\ y^{t}=\sigma \left(w^{\prime }h^{t}\right)\text{.} \end{array}$$

The calculation of the output results can indicate the data information that LSTM needs to focus on memorizing, that is, LSTM can decide to eliminate useless information through the calculation results, thereby retaining useful information. LSTM and RNN technology also have forward output and reverse error transmission, so it is necessary to calculate its weight derivative, as shown in:

(4) $$\begin{array}{c} \delta_{j}^{t}≜\frac{\partial O}{\partial a_{j}^{t}}\text{,} \end{array}$$

*O* means the loss function and *∂* indicates the partial derivative. By this forward calculation, the calculation of the input gate is as follows:

(5) $$\begin{array}{c} a_{l}^{t}=\overset{I}{\underset{i=1}{\sum }}w_{il}x_{i}^{t}+\overset{H}{\underset{h=1}{\sum }}w_{hl}b_{h}^{t-1}+\overset{C}{\underset{c=1}{\sum }}w_{cl}s_{c}^{t-1}\text{.} \end{array}$$

The forget gate is calculated as

(6) $$\begin{array}{c} a_{\phi }^{t}=\overset{I}{\underset{i=1}{\sum }}w_{i\phi }x_{i}^{t}+\overset{H}{\underset{h=1}{\sum }}w_{h\phi }b_{h}^{t-1}+\overset{C}{\underset{c=1}{\sum }}w_{c\phi }s_{c}^{t-1}\text{.} \end{array}$$

The calculation of the memory cell is

(7) $$\begin{array}{c} a_{c}^{t}=\overset{I}{\underset{i=1}{\sum }}w_{ic}x_{i}^{t}+\overset{H}{\underset{h=1}{\sum }}w_{hc}b_{h}^{t-1}\text{,}\\ s_{c}^{t}=b_{\phi }^{t}s_{c}^{t-1}+b_{l}^{t}g\left(a_{c}^{t}\right)\text{.} \end{array}$$

The computation of the output gate is written in equations (8) and (9):

(8) $$\begin{array}{c} a_{\psi }^{t}=\overset{I}{\underset{i=1}{\sum }}w_{iy}x_{i}^{t}+\overset{H}{\underset{h=1}{\sum }}w_{h\psi }b_{h}^{t-1}+\overset{C}{\underset{c=1}{\sum }}w_{a\psi }s_{c}^{t-1}\text{,} \end{array}$$

(9) $$\begin{array}{c} b_{\psi }^{t}=f\left(a_{\psi }^{t}\right)\text{.} \end{array}$$

If it is reversed, the calculation of the unit output is as follows:

(10) $$\begin{array}{c} \varepsilon_{c}^{t}=\overset{K}{\underset{k=1}{\sum }}w_{ck}\delta_{k}^{t}+\overset{H}{\underset{h=1}{\sum }}w_{ch}\delta_{h}^{t+1}\text{.} \end{array}$$

Equation (11) represents the calculation of the output gate:

(11) $$\begin{array}{c} \varepsilon_{\psi }^{t}=f^{\prime }\left(a_{\psi }^{t}\right)\overset{c}{\underset{c=1}{\sum }}h\left(s_{c}^{t}\right)\varepsilon_{k}^{t}\text{.} \end{array}$$

The equation for calculating the current state is

(12) $$\begin{array}{c} \varepsilon_{s}^{t}=b_{\psi }^{t}h^{\prime }\left(s_{c}^{t}\right)\varepsilon_{c}^{t}+b_{\phi }^{t+1}\varepsilon_{s}^{t+1}+w_{cl}\delta_{l}^{t+1}+w_{c\phi }\delta_{\phi }^{t+1}+w_{\alpha \nu }\delta_{w}^{t}\text{.} \end{array}$$

The calculation of memory unit is indicated in:

(13) $$\begin{array}{c} \delta_{c}^{t}=b_{l}^{t}g^{\prime }\left(a_{c}^{t}\right)\varepsilon_{c}^{t}\text{.} \end{array}$$

Equation (14) displays the computation of the forget gate:

(14) $$\begin{array}{c} \delta_{\phi }^{t}=f^{\prime }\left(a_{\phi }^{t}\right)\overset{c}{\underset{c=1}{\sum }}s_{c}^{t-1}\varepsilon_{s}^{t}\text{.} \end{array}$$

The following is the calculation equation of the input gate:

(15) $$\begin{array}{c} \varepsilon_{l}^{t}=f^{\prime }\left(a_{l}^{t}\right)\overset{c}{\underset{c=1}{\sum }}g\left(a_{c}^{t}\right)\varepsilon_{s}^{t}\text{.} \end{array}$$

The LSTM-based deformation prediction model of the building envelope is constructed, evaluated, and analyzed. This model mainly calculates the condition of the envelope structure through the LSTM algorithm and then predicts the deformation result of the envelope structure. It has the advantage of being able to perform the cyclic calculation to reduce the model's prediction error and improve the prediction accuracy of the deformation of the building envelope.

### 2.4. Experimental Data and Parameter Settings

The main research purpose is to predict the deformation of the envelope structure of underground buildings based on the LSTM model. The data studied come from the observation data of the deformation of the envelope structure at the settlement monitoring point of the foundation pit column of a subway in Chengdu and a total of 80 observation periods. First, the abnormal data in the detection data are extracted, 60 periods of data in the data are used as the model's training data, and the remaining 20 periods are used as the detection data of the model. In the prediction process, models with different training times are used as the calculation model, to understand the comprehensive performance of the model more clearly. A total of six groups of models are set up, and the training times are 10, 20, 30, 40, 50, and 60 times, respectively, to explore the comprehensive performance of the model under different training times.  Table 1 shows the observation data of 80 periods.

## 3. Research Results

### 3.1. Deformation Analysis of Building Envelope under DL Technology

Based on DL technology, it designs and uses LSTM algorithm to predict the deformation of the underground building envelope, to improve the safety of it and promote the comprehensive development of the underground building industry.  Figure 4 indicates the prediction results of the displacement of the diaphragm wall foundation pit pile using the LSTM algorithm.

In Figure 4(a), the training times are 10–60 times, respectively, and the horizontal displacement measurement values of the pile body of the diaphragm wall foundation pit under different periods are counted.  Figure 4(b) is the mean relative error (MRE) value and calculation time of the model under different training times under the horizontal displacement of the pile body.  Figure 4(c) displays the pile settlement distance under different periods and different training times.  Figure 4(d) is the MRE value and calculation time of pile settlement for different training times. The designed LSTM algorithm model can relatively accurately predict the pile displacement of the diaphragm wall foundation pit. In the prediction of the horizontal displacement of the pile, according to the comparison of different periods, it is found that the prediction accuracy of the designed LSTM algorithm model increases with the number of training increases. The MRE of prediction results of the model is around 18% at the highest and around 10% at the lowest. The calculation time of the model will become relatively stable as the number of training increases, and the gap generated during the prediction process is small. The longest prediction time is about 36 s, and the shortest is about 15 s. In the prediction of the settlement and displacement of the pile, the prediction results of the designed model are also very satisfactory. As the number of training increases, the accuracy of the prediction results also increases. The MRE of the model's prediction results is about 7% at the highest and about 5% at the lowest. Similarly, the calculation time of the model will become relatively stable as the number of training increases, with the longest calculation time being around 40 s and the shortest being around 17 s.

### 3.2. Performance Analysis of Models by DL Technology

The LSTM algorithm model is designed by using DL technology, and the comprehensive performance of the model is analyzed, but its advantages in the current industry have not yet been reflected. Therefore, to comprehensively reflect the performance advantages of this model, the designed LSTM model and other models are compared. The comparative results of the relative error of the deformation analysis of the building envelope between the designed model and other models are illustrated in Figure 5.

In Figure 5, the deformation analysis of the underground building envelope between the designed model and other models illustrates that the relative error of the predicted results of the designed model is about 5.4% at the highest and 1.8% at the lowest. The lowest of other models is around 5.4%, and the highest is around 13.1%. It means that the performance of the designed LSTM model is better than other models.

## 4. Conclusion

With the growth of urban architecture, to reduce the excessive occupation of land by above-ground buildings, underground buildings have become one of the mainstream architectural forms. The safety assurance of these buildings is relatively difficult. To improve the current dilemma of safety analysis of such buildings, the underground building envelope is first discussed, and then the DL technology and the basic concept of the LSTM model are expounded. At last, the LSTM displacement prediction model is designed on account of the safety prediction of the underground building envelope, and the model is comprehensively evaluated. The findings manifest that in the evaluation of the horizontal displacement of the pile, the prediction accuracy of the designed LSTM algorithm model increases with the training increases, and the MRE of the model's prediction results is about 18% at the highest. The calculation time of the model will become relatively stable with the increase of training times, and the gap generated in the prediction process is small, and the shortest prediction time is about 15 s. In the prediction of the settlement and displacement of the pile, the overall model with the increase of training times, the accuracy of the prediction results also increases relatively, and the MRE of the model's prediction results is about 7% at the highest. Similarly, the calculation time will become relatively stable with the increase of the number of training, among which the calculation time is the shortest around 17 s. Compared with other models, it is found that the relative error of the prediction results of this model is about 5.4% at the highest and 1.8% at the lowest. Although the comprehensive prediction performance comparison results of the models are provided, the practical application of the model is not enough, so the comprehensive research on the practical application of the model will be strengthened in the future. The deformation value of the envelope structure in the later stage is predicted, and the deformation trend is predicted in time. When the deformation of the deep foundation pit exceeds the allowable range of deformation, the protection scheme can be taken in time to effectively reduce the casualties and economic losses caused by accident. This exploration provides technical support for deformation analysis of underground building envelopes and provides a reference for safety analysis and optimization of underground buildings.

## Figures and Tables

**Figure 1:** The basic principle of the composite envelope of a diaphragm wall and multiple rows of steel plates ((a) refers to the composite envelope of a diaphragm wall and multiple rows of steel plates, (b) indicates the traditional building envelope).

**Figure 2:** Methods of reinforcement of the composite envelope by the diaphragm wall ((a) the reinforcement of advance precipitation in the pit, (b) the reinforcement of high-pressure jet grouting, (c) the reinforcement of cement-soil mixing, and (d) the grouting reinforcement).

**Figure 3:** The comparison effect of LSTM and common RNN techniques and the working principle of LSTM ((a) the common RNN technology; (b) the basic composition of LSTM; (c) the working principle of LSTM).

**Figure 4:** The prediction results of the displacement of the diaphragm wall foundation pit pile ((a) means the prediction of the horizontal displacement of the pile, (b) signifies the analysis of the prediction of the horizontal displacement of the pile, (c) shows the prediction of the settlement of the pile, and (d) manifests the analysis of the prediction of the settlement of the pile).

**Figure 5:** The comparative results of the relative error of the deformation analysis of the building envelope between the designed model and other models.

**Table 1:** Monitoring data statistics.

Period	Observed value/mm	Period	Observed value/mm	Period	Observed value/mm	Period	Observed value/mm
1	−0.44	21	−0.04	41	−0.5	61	17.57
2	−0.68	22	−0.61	42	−0.7	62	20.51
3	−0.92	23	−0.82	43	−0.78	63	18.88
4	−0.88	24	−0.79	44	−0.75	64	18.98
5	−0.66	25	−0.59	45	−0.58	65	19.94
6	−0.95	26	−0.85	46	−0.8	66	17.28
7	−0.88	27	−0.79	47	−0.75	67	19.73
8	−0.75	28	−0.67	48	−0.65	68	18.24
9	−0.68	29	−0.61	49	−0.6	69	20.91
10	0.12	30	0.09	50	0.07	70	21
11	0.42	31	−0.45	51	−0.39	71	17.53
12	−0.65	32	−0.58	52	−0.61	72	18.41
13	−0.84	33	−0.98	53	−0.81	73	20.75
14	−0.99	34	−0.87	54	−0.78	74	19.03
15	−0.73	35	−0.56	55	−0.59	75	17.97
16	−0.86	36	−1.04	56	−0.84	76	19.27
17	−0.81	37	−0.82	57	−0.78	77	18.06
18	−0.7	38	−0.85	58	−0.67	78	17.89
19	−0.65	39	−0.72	59	−0.61	79	20.58
20	−0.08	40	0.07	60	0.1	80	20.66

## Data Availability

All data are fully available without restriction.
